The article "Antibody development for preventing the human respiratory syncytial virus pathology" was published in 2020. Journal: Mol Med.

# Antibody development for preventing the human respiratory syncytial virus pathology

**DOI:** 10.1186/s10020-020-00162-6

**Published:** 2020-04-17

**Authors:** Jorge A. Soto, Nicolás M. S. Gálvez, Gaspar A. Pacheco, Susan M. Bueno, Alexis M. Kalergis

**Affiliations:** 1 Millennium Institute on Immunology and Immunotherapy, Departamento de Genética Molecular y Microbiología, Facultad de Ciencias Biológicas, Pontificia Universidad Católica de Chile, Avenida Libertador Bernardo O’Higgins #340, 8331010 Santiago, Chile; 2 Departamento de Endocrinología, Facultad de Medicina, Pontificia Universidad Católica de Chile, Santiago, Chile

**Keywords:** hRSV, Human orthopneumovirus, Antibodies, Therapy, Prophylaxis, Passive transference

## Abstract

Human respiratory syncytial virus (hRSV) is the most important etiological agent causing hospitalizations associated with respiratory diseases in children under 5 years of age as well as the elderly, newborns and premature children are the most affected populations. This viral infection can be associated with various symptoms, such as fever, coughing, wheezing, and even pneumonia and bronchiolitis. Due to its severe symptoms, the need for mechanical ventilation is not uncommon in clinical practice. Additionally, alterations in the central nervous system -such as seizures, encephalopathy and encephalitis- have been associated with cases of hRSV-infections. Furthermore, the absence of effective vaccines or therapies against hRSV leads to elevated expenditures by the public health system and increased mortality rates for the high-risk population. Along these lines, vaccines and therapies can elicit different responses to this virus. While hRSV vaccine candidates seek to promote an active immune response associated with the achievement of immunological memory, other therapies -such as the administration of antibodies- provide a protective environment, although they do not trigger the activation of the immune system and therefore do not promote an immunological memory. An interesting approach to vaccination is the use of virus-neutralizing antibodies, which inhibit the entry of the pathogen into the host cells, therefore impairing the capacity of the virus to replicate. Currently, the most common molecule targeted for antibody design against hRSV is the F protein of this virus. However, other molecular components of the virus -such as the G or the N hRSV proteins- have also been explored as potential targets for the control of this disease. Currently, palivizumab is the only monoclonal antibody approved for human use. However, studies in humans have shown a protective effect only after the administration of at least 3 to 5 doses, due to the stability of this vaccine. Furthermore, other studies suggest that palivizumab only has an effectiveness close to 50% in high-risk infants. In this work, we will review different strategies addressed for the use of antibodies in a prophylactic or therapeutic context and their ability to prevent the symptoms caused by hRSV infection of the airways, as well as in other tissues such as the CNS.

## Introduction

Human respiratory syncytial virus (hRSV), recently re-named human orthopneumovirus (Afonso et al. 2016), is the main virus responsible of respiratory diseases in newborns, children under 5 years old, and the elderly. hRSV is the most important viral agent causative of acute lower respiratory tract infections (ALRTI) and hospitalizations during winter season (Nair et al. 2010). The symptoms associated with the infection of this virus are mostly age-dependent (Domachowske et al. 2018a), although they are frequently related to coughing, wheezing, fever, apnea, and bronchiolitis or pneumonia in some cases. Commonly, afflicted children require supportive care, accompanied with supplemental oxygen and, in extreme cases, the use of mechanical ventilation (Krilov 2011). Remarkably, extrapulmonary symptoms have also been described for this disease, including cardiovascular complications in young infants (Gálvez et al. 2017; Puchkov and Min’kovich 1972; Suda et al. 1993; Donnerstein et al. 1994), hepatitis -associated with liver complications- (Gálvez et al. 2017; Eisenhut and Thorburn 2002; Eisenhut et al. 2004), hyponatremia (Hanna et al. 2007) and alterations in the central nervous system (CNS), such as seizures (Cha et al. 2019), encephalopathy and encephalitis (Bohmwald et al. 2015). Additionally, hRSV infections can result in impaired learning capacities, as described in murine models (Gálvez et al. 2017; Bohmwald et al. 2018; Espinoza et al. 2013). Accordingly, symptoms such as apnea, encephalopathy, seizures, strabismus and status epilepticus have also been reported in humans (Sweetman et al. 2005; Kho et al. 2004; Millichap and Wainwright 2009; Kawashima et al. 2012), adding to the long list of collaterals from this disease. Further studies analyzing the disease induced by this virus are still required to elicit its true impact as a possible systemic pathogen and the new relevance that this could have from a clinical perspective.

hRSV is associated with a rate of infection close to 34 million children under 5 years old per year (Bont et al. 2016). Specifically, hRSV is responsible of nearly 63% of total ALTRI cases and between 19 to 81% of the total viral infections affecting the lower respiratory tract in children. This wide range indicated above is associated with a retrospective analysis that covered 20 years of epidemiology data (Bont et al. 2016). One out of ten children infected with hRSV is hospitalized due to the severe symptoms induced by this virus, and the World Health Organization has estimated that 66,000 to 253,000 annual deaths are due to hRSV (Afonso et al. 2016; Bont et al. 2016). Finally, children hospitalizations due to hRSV-related bronchiolitis can even reach an 80% in the USA (Peiris et al. 2003).

hRSV was first isolated and identified the year 1956 from a colony of chimpanzees (Chanock and Finberg 1957). Recently, hRSV was reclassified as a member of the *Orthopneumovirus* genus and *Pneumoviridae* family (Afonso et al. 2016). Its viral genome consists of a single-stranded (ss) and negative-sensed (−) RNA, composed of 15.2 Kb with 10 genes that codify for 11 proteins, including two non-structural proteins (NS) and nine structural proteins, translated in the following order 3′- NS1-NS2-N-P-M-SH-F-G-M2.1-M2.2-L- 5′ (Gálvez et al. 2017; Hacking and Hull 2002).

Once hRSV reaches its host, it is able to infect the respiratory tract, mainly targeting epithelial cells at the alveolar epithelium. Here, the glycoprotein (G) is anchored to the plasmatic membrane of its target cell. Then, the fusion protein (F) promotes the fusion between the viral envelope and the plasmatic membrane of the host cell. The fusion process allows the entry of the genetic material that can be used for replication and transcription, once the replicase/transcriptase complex (conformed by the N-, P-, and L- hRSV proteins) is assembled (Hacking and Hull 2002; Collins and Melero 2011). Other viral proteins, such as M2.1 and M2.2, are used as cofactors for this replicase/transcriptase complex (Harpen et al. 2009). The genome is replicated into a positive-sensed (+) antigenome, which will be used for the generation of new genetic material. In parallel, the viral genome will be transcribed into a (+) mRNA, that will be used for protein synthesis (Hacking and Hull 2002). All these processes results in the synthesis of a new ssRNA (−) genome, that will eventually be used as a template for the synthesis of new proteins by the host’s ribosomes (Hacking and Hull 2002; Collins and Melero 2011; Tsutsumi et al. 1995) originating new viral particles after 10–12 h post cell infection (Collins and Karron 2013).

Both non-structural proteins -NS1 and NS2- are virulence factors with a key role in the immune evasion mechanisms and the induction of cellular apoptosis elicited by hRSV, undermining the host’s defenses (Liesman et al. 2014; Lo et al. 2005; Pretel et al. 2013). Specifically, NS1 and NS2 have been associated with the suppression of the type I IFN pathway, by impairing the regulation of STAT2. As a consequence, both downstream α/β IFN genes are suppressed leading to an inefficient viral clearance by the host (Lo et al. 2005; Pretel et al. 2013). Additionally, NS2 has been associated with the obstruction of the airways, as it promotes the shedding of epithelial cells into the airways (Liesman et al. 2014). Therefore, both non-structural proteins contribute to the suppression of type I IFN secretion, which is one of the host’s first line of defense for the elimination of viral pathogens.

To control the disease caused by hRSV, several vaccines and treatments were developed soon after its discovery (WHO PD-VAC 2014; Graham 2016; Modjarrad et al. 2016). However, no convincing results -both regarding safety and immunogenicity- have been obtained after the numerous vaccine trials that may allow approving the use of a vaccine in humans (Graham 2016). One of the first vaccines tested for hRSV was a formalin-inactivated virus vaccine (FI-hRSV), a formulation that exacerbated the detrimental inflammatory response triggered by the virus in infants and regrettably ended up with the death of two of the immunized children (KIM et al. 1969; Murphy and Walsh 1988). In this line, recent reports have indicated that differential subsets of CD4^+^ T cells are responsible of the exacerbated response elicited by this failed vaccine prototype (Knudson et al. 2015). In order to control hRSV’s expansion worldwide in a safer way, prophylactic approaches based on anti-hRSV antibodies have been generated. These molecules are generally known to be less immunogenic and hold an acceptable safety record for the control of microbial pathogens.

There are significant differences between the development of vaccines versus antibody-based prophylactic therapies, especially for a pathogen such as hRSV (Wang et al. 2019; Villafana et al. 2017; Simões et al. 2018). Although the main aim of both types of treatment is to achieve a protective response against the virus, active immunization with vaccines usually results in the activation and generation of immunological memory by the adaptive immune response. Antibody-based prophylactic are preventive strategies that usually promote a protective response that does not lead to the activation of the immune system, nor the induction of immunological memory. This type of immune protection relies on the periodic administration of pathogen-specific antibodies and depends on the half-lives of these molecules (Baxter 2007). The antibody-based prophylaxis and other related preventing therapies developed up to date against hRSV will be discussed in the following sections.

### Antibody-based approaches for hRSV for high-risk populations

Following the discovery of hRSV, the development of vaccines and treatments was quickly initiated (Fig. 1). After the detrimental effects elicited by the FI-hRSV vaccine in children (2 months to 9 years) (KIM et al. 1969; Chin et al. 1969), the notion of a prophylactic treatment based on the passive transfer of hRSV-specific antibodies was supported by early studies and reports in cotton rats (Prince et al. 1985). The results showed therein considered an extensive description of the properties of these antibodies, such as opsonization, neutralization and the capacity to induce clearance of some pathogenic agents. This work was considered a starting point for the use of antibodies as a new tool against hRSV (Olszewska and Openshaw 2009). Early studies generated and evaluated almost 25 different hybridomas, used to obtain several anti-P, −N, −G and -F antibodies (Fig. 1) (Stott et al. 1984). The authors of this work indicated that optimal results were obtained only for one anti-F and one anti-G antibody in mouse model (Taylor and Stott 1984). However, one of the most critical caveats of these antibodies was their low neutralizing capacity in murine models. An encouraging discovery of these studies was the identification of specific sites on the F- and G-hRSV proteins that promote the binding of monoclonal antibodies with enhanced neutralizing capacity (Anderson et al. 1986).

**Fig. 1:** Timeline of antibodies therapies since the discovery of hRSV as human pathogen. Advances and implementation of different strategies that use antibodies to promote the clearance of hRSV since the virus was first discovered in 1956

The use of Intravenous Immunoglobulin (IVIG), a pool of polyclonal antibodies, was another therapy utilized at one point to prevent lethal hRSV infections in high-risk populations (Fig. 1). In preterm infants and children with cardiac diseases, different doses of IVIG with specificity against hRSV (IVIG-hRSV) were tested (150 mg/kg to 750 mg/kg) and only the highest IVIG-hRSV dose tested elicited a significant protection. The highest IVIG-hRSV dose decreased the hospitalization days, ameliorated the symptoms and reduced the number of ALRTI cases, when compared to the lower doses and the placebo-treated control groups (Groothuis et al. 1993). A similar study evaluated a total of 510 children either premature at birth or with cardiac diseases. This study showed that monthly administration of both the low and the high IVIG-hRSV doses resulted in beneficial effects, as compared to placebo controls or to children receiving a single dose (Groothuis et al. 1993). These results were independent of the pathology or the recurrence in the development of the respiratory diseases, as compared with the children treated with the low dose or the placebo control groups (Respiratory Syncytial Virus (RSV) PREVENT study group 1997). Importantly, the use of IVIG-hRSV as a therapy (RespiGam, Massachusetts Public Health Biologic Laboratories, and MedImmune, Inc., Gaithersburg, MD.) was approved by the Food and Drug Administration (FDA) in 1996 for hRSV’s high risk populations (Committee on Fetus and Newborn 2004).

Soon after the approval of RespiGam by the FDA, a humanized IgG1-isotype monoclonal antibody against the F-hRSV protein was produced and baptized as MEDI-493 or palivizumab. Currently, this antibody is the only prophylactic therapy approved and used in high-risk populations to treat and prevent hRSV infections (Simões et al. 2018). Since it showed a greater protective effect than IVIG, the FDA decided to keep it as the only therapy approved (Johnson et al. 1997). Despite this, two other antibodies against the F-hRSV protein, generated by Merck and Sanofi, are currently undergoing Phase I and III clinical trial evaluations, respectively. Interestingly, targeting the N-hRSV protein has been considered as a new approach, as this protein can be found on the surface of hRSV-infected cells (Cespedes et al. 2014). It is thought that anti-N-hRSV antibodies might lead to the killing of infected cells preventing virus spread, as it will be discussed below.

### Production of an anti-G monoclonal antibody as an improved immunotherapy against hRSV

One of the first monoclonal antibodies developed after the IVIG-hRSV was an anti-G-hRSV antibody (131-2G) that only exhibited partial neutralization capacities (Anderson et al. 1988). This monoclonal antibody blocks the interaction between the G protein and the CX3C chemokine receptor by recognizing a conserved epitope on the G protein that is required for binding to its receptor (Tripp et al. 2001; Tripp et al. 2003). Although in vitro studies using the 131-2G antibody showed reduced neutralization capacity, in vivo responses showed activation of Fc receptors and a better protective response than others anti-F monoclonal antibodies (Radu et al. 2010; Miao et al. 2009). The pathology induced upon hRSV infection was also decreased when the 131-2G antibody was administered, correlating its neutralizing capacity with a lower pulmonary inflammatory disease (Miao et al. 2009; Haynes et al. 2009). Interestingly, a protective response was observed even when the antibody was administered 5 days after the infection (Haynes et al. 2009).

While the native 131-2G monoclonal antibody was able to favor the development of a Th1-like immune response, inducing the secretion of IFN-γ, a modified version of this antibody consisting of only the F(ab’)_2_ region promoted a Th2-like profile, without an optimal viral clearance (Boyoglu-Barnum et al. 2014). Despite these promising data, to date no further evaluation of this antibody in clinical studies has been published.

The 131-2G antibody was also tested along with another anti-G monoclonal antibody (130-6D) that recognizes an epitope located at the central conserved region (CCR) of the G-hRSV protein. In this study, authors showed that the combination of both monoclonal antibodies decreased the lung pathology when compared to the administration of solely the 130-6D monoclonal antibody, without affecting their mutual neutralization effects (Caidi et al. 2012).

### Palivizumab: a passive prophylactic method to protect against hRSV infection

Palivizumab (MEDI-493, Synagis, MedImmune, Inc., Gaithersburg, MD) is a commercially distributed, humanized IgG1 monoclonal antibody that binds to the F-hRSV protein (Johnson et al. 1997). The first study that described the effect of palivizumab in vivo was performed in cotton rats treated 1 day prior to hRSV infection showing a decrease in the disease parameters when compared to the control (Johnson et al. 1997). Of these results two possible mechanisms arose to understand the palivizumab activity. First, palivizumab is able to prevent the fusion between the viral particle and the host cell membrane and second, it might suppress the formation of syncytia between lung epithelial cells, effect observed in lung epithelial cells in vitro. These could be achieved by blocking the interaction between the F protein and the proteins found at the host cell surface (Young 2002).

Following the experiments performed in animal models, clinical studies were performed for palivizumab (Subramanian et al. 1998; Sáez-Llorens et al. 1998). These studies showed that a monthly administration of this antibody was necessary to decrease the disease parameters in the population evaluated, and that this dosage maintained the monoclonal antibody detectable up until day 30 post-immunization in the serum (Subramanian et al. 1998; Sáez-Llorens et al. 1998). The use of palivizumab was also tested as therapy in children hospitalized due to an hRSV infection. Interestingly, a decrease in number of plaque-forming units (PFU) in children treated with palivizumab when compared to the placebo-treated controls was found. However, the observed decrease in PFUs did not correlate with any change in the cellular immune responses (DeVincenzo et al. 2007). In addition, palivizumab administration promoted a reduction in the number of hospitalizations of this high-risk population. The children treated with palivizumab exhibited shorter hospitalization periods and a decreased requirement of oxygen assistance, along with a less pronounced development of ALRTI than the untreated control groups (Village 1998).

The main caveat of palivizumab is the very high cost/effectiveness ratio, since as many as 5 doses might be needed to decrease the probability of a potent or lethal hRSV infection in a high-risk population, given the half-life of the antibody in the host (Village 1998; B. R. 2018; Torchin et al. 2018). The elevated cost for completing an effective treatment is a major burden for health care programs (US$780 per vial of 50 mg and US$1416 per vial of 100 mg, with a recommended dosage of 15 mg/kg) (Ambrose et al. 2014; Mochizuki et al. 2017). The need of multiples doses reflects the inability of palivizumab to induce a long-lasting immune protection in the individual, therefore consisting of a passive immunization treatment.

Finally, some weak points associated with the use of palivizumab are that both dosage and periodicity of administration can influence the effectiveness of the treatment (B. R. 2018). Besides, it suggested that children previously exposed to palivizumab exhibited more respiratory problems than children exposed to this antibody for the first time. Nevertheless, the authors of the study suggested that these respiratory problems might not be associated directly to palivizumab, but rather to environmental factors (Lacaze-Masmonteil et al. 2003).

### Motavizumab, an improved version of palivizumab

Motavizumab (MEDI-524) is an improved version of palivizumab, with an optimized affinity for the F-hRSV protein achieved by mutating 13 specific amino acids located in the variable region of the Complementary Determining Region (CDR) sequence of the antibody (Wu et al. 2007; Wu et al. 2008). Early data derived from the use of motavizumab showed a 70-fold increase in binding to the F-hRSV protein as compared to palivizumab. Interestingly, motavizumab was able to decrease the infection in the upper respiratory tract in a cotton rat model, an effect that was not observed when palivizumab was used as a treatment instead (Wu et al. 2007; Mejías et al. 2005).

The suggested mechanism of action of motavizumab as a novel therapy is the inhibition of the cell-to-cell fusion, without affecting the attachment of the virus to the target cell. The central hypothesis surrounding this suggested mechanism considers the antibody’s capacity of interrupting the conformational change of the F protein at the moment of making the fusion with the cell membrane of the host cell, therefore targeting the pre- and- post-fusion F protein (Huang et al. 2010).

A Phase II clinical study evaluated the effect of five-administrations of either: motavizumab only, motavizumab and then palivizumab (M/P), or palivizumab and then motavizumab (P/M). As expected, the three groups showed a similar protective response. However, when comparing the adverse events (AEs) induced by these treatments, the highest AEs incidence was reported for the M/P-treated children. Although two deaths were reported for the M/P group, according to the authors the deaths and the pulmonary impairment reported were not associated with the treatment (Fernández et al. 2010).

A phase III clinical trial for motavizumab was also performed in children under 6 months old, which were treated with this antibody and their response was compared to that of children treated with palivizumab (Carbonell-Estrany et al. 2010). The authors observed that there were less cases of hospitalization among children treated with motavizumab than among those treated with palivizumab (Carbonell-Estrany et al. 2010). These data suggested that motavizumab is a more efficient prophylactic treatment than palivizumab. However, these motavizumab-treated children exhibited more frequent AEs, specifically associated with cutaneous problems, such as rashes and skin-related allergies (Carbonell-Estrany et al. 2010).

Another phase III clinical trial was performed in a population of 2596 children, either preterm (born at 36 weeks) or under 6 months of age (O’Brien et al. 2015). A positive protective effect was shown for motavizumab for both inpatient and outpatient burdens. This study also demonstrated that children treated with motavizumab exhibited less severe hRSV infections and achieved a reduction in hospitalization rates and in the need of mechanical ventilation, when compared to placebo-treated groups (O’Brien et al. 2015). This study corroborated observations reported previously, indicating that motavizumab elicits an enhanced protective capacity against hRSV-infections, when compared to palivizumab (Carbonell-Estrany et al. 2010; O’Brien et al. 2015).

Despite of all the positive findings made with motavizumab, a phase II clinical trial that analyzed a population of 118 children showed that the use of two different doses of motavizumab was not able to significantly decrease viral loads in treated children (Ramilo et al. 2014). Furthermore, lack of reduction in viral loads was associated with the absence of improvement of treated children (Ramilo et al. 2014). The following of these children for 12 months after the treatment showed equivalent rates of wheezing episodes as compared to the controls (Ramilo et al. 2014). Interestingly, the vast majority of studies using antibody therapies in humans have shown that this type of transfer is not capable of directly decreasing viral loads in the subjects (Millichap and Wainwright 2009; Bont et al. 2016; Tsutsumi et al. 1995).

Unfortunately, despite motavizumab’s higher efficiency as a therapy against hRSV, the FDA decided not to approve the license for this new antibody and decline to endorse an extensive use in humans. This decision was based on the large number of AEs associated to skin allergies reported in the clinical study of Carbonell-Estrany et al. described above (Carbonell-Estrany et al. 2010).

### Development of mucosal antibodies-based strategies as a prophylaxis for hRSV

As hRSV-infections are mainly associated with the respiratory tract (Nair et al. 2010), the development of strategies focused on mucosal antibodies could improve the treatment of the disease caused by this pathogen. Antibodies are categorized-according to the characteristics of their Fc domain as IgM, IgG, IgD, IgE and IgA (Mak et al. 2014). The IgA isotype is especially important as it constitutes one of the first mucosa defense barriers against various infectious agents (Woof and Russell 2011). An early study showed that the intranasal administration of an anti-F-hRSV mouse monoclonal IgA antibody (HNK20) -prior to hRSV infection- reduced viral titers in the lungs both in mice and rhesus monkeys (Weltzin et al. 1994; Weltzin et al. 1996). Despite these encouraging data in animal models for this HNK20 antibody, a phase III clinical trial showed unconvincing results and a further development of this antibody was not pursued (Mills et al. 1999).

A recent study used the Fab regions of palivizumab and motavizumab to generate recombinant monomeric, dimeric and secretory IgA molecules (Jacobino et al. 2018). The main particularity of these molecules was their capacity to recognize the same epitopes as palivizumab and motavizumab but displaying the functional features of an IgA molecule. Such isotype change resulted in a decrease effectivity of these recombinant IgA antibodies, as compared to the IgG1 palivizumab and motavizumab (Jacobino et al. 2018). Reduced in vitro and in vivo antiviral responses in the mouse model also discouraged further studies for these recombinant IgA molecules (Jacobino et al. 2018).

However, it is important to mention that various studies in adult populations have reported high titers of IgA and IgG antibodies, mainly against the G- and the F-hRSV proteins (Cortjens et al. 2017; Goodwin et al. 2018). In a study performed by Cortjens et al., the effect and isotype of antibodies produced by isolated memory B cells from healthy donors was evaluated. These memory B cells were used for the generation of hybridomas whose secreted antibodies were evaluated in hRSV-infected cells. However, these antibodies exhibited limited neutralizing capacity, a signature of hRSV-induced antibodies, as this virus is responsible of recurrent viral infections throughout the life (Cortjens et al. 2017).

IgA has even been suggested as a possible predictor of hRSV-infection susceptibility after a study with a cohort of 61 healthy volunteers (Habibi et al. 2015). Despite the negative results and the reduced number of researches focusing on the development of IgA antibodies as a therapy for hRSV, a study using monoclonal IgA and IgG isotype antibodies against Influenza virus showed that IgAs can promote better prevention of viral infections as compared to IgGs (Muramatsu et al. 2014).

A summary of the current advances and the most important developments of antibodies used as therapies are described in Fig. 2, where the main features of each treatment are highlighted.

**Fig. 2:** Development of antibody therapies against hRSV infection. The five main types of antibody therapies against the hRSV-infection are described. Also, these therapies are shown in order of development, highlighting that the only approved therapy to be used in humans to date is palivizumab. However, an interesting new possibility is also described at the end of the figure, associated with a therapy based on the use of the monoclonal anti-N-hRSV antibody

### Novel hRSV antigen targets for the design of protective antibodies

Currently, there are only a few monoclonal antibodies conceived as a prophylactic treatment under development. Three preclinical candidates have been published on the Program for Appropriate Technology in Health (PATH website). Two of these antibodies recognize the F-hRSV protein (Arsanis and UCAB (mAbXience)), and one of them is specific for the N-hRSV protein. The anti-N antibody was first evaluated in clinical samples from nasopharyngeal swabs obtained from patients infected with hRSV, showing a high specificity for this protein (Gómez et al. 2014). The protective capacity of this antibody -which is currently under preclinical evaluation in animal models- is based on the induction of an antibody dependent cell cytotoxicity (ADCC) of hRSV-infected cells. As the N-hRSV protein can be found on the surface of infected cells (Cespedes et al. 2014), an anti-N-hRSV antibodies could induce ADCC and complement fixation on cells infected with hRSV. This antibody is yet to be evaluated in humans.

The rationale of using an anti-N-hRSV antibody relies on the capacity of this protein to migrate to the membrane of infected cells (Cespedes et al. 2014) and the consequent impairment of the immunological synapses reported (Cespedes et al. 2014). It is possible that the recently described feature of the N-hRSV protein could contribute on preventing the establishment of an adequate immunological synapse, required for the proper induction of a protective Th1 response, during an hRSV infection. Therefore, the use of this antibody could contribute to restore the induction of the cytotoxic immune response required to clear this virus.

As stated above, two novel antibodies are currently undergoing clinical evaluation with the F-hRSV protein as their target (Aliprantis et al. 2018; Zhu et al. 2017). The first one is known as MK-1654, a human monoclonal antibody that possess a modification in the Fc region to promote an increase in the molecule half-life (Aliprantis et al. 2018). MK-1654 was developed by Merck™, and the target group for administration are the pediatric population. Currently, this antibody is being evaluated in a clinical trial (Aliprantis et al. 2018). The second anti-F-hRSV antibody (MedImmune, Sanofi) called MEDI8897 is a recombinant human IgG1 monoclonal antibody that recognizes the pre-fusion state of the F-hRSV protein. The pre-fusion state of the F-hRSV protein is a metastable homotrimer associated to type I fusion proteins of different viruses. A conformational change occurs after an initial cleavage of the inactive precursor of the F-protein (F0). Then, after the fusion between the host membrane and the viral membrane, the F-hRSV protein adopts a stable post-fusion conformation (Magro et al. 2010; Ngwuta et al. 2015; McLellan et al. 2011). A study performed in cotton rats showed a 9-fold increase in the reduction of viral loads in the lungs of infected animals, when compared to animals receiving palivizumab (Zhu et al. 2017). A clinical study using MEDI8897 in a dose-escalated study showed that a single dose of this antibody in healthy preterm infants promoted a safe response with neutralizing capacity at its highest dose (50 mg) (Domachowske et al. 2018b). Another clinical trial using the same antibody previously confirmed safety in healthy adults (Griffin et al. 2017). Currently this antibody is being evaluated in a phase III trial.

Despite the similarities between many of these antibodies in their structure (and possibly, their function), when they are evaluated as a treatment, minimal changes might be critical to promote protection. Some of the main advantages and disadvantages of the above discussed monoclonal antibodies are shown in Table 1.

**Table 1:** Advantages and disadvantages of several antibodies against hRSV-infection

Name	Target/Type	Advantages	Disadvantages	Reference
IVIG-hRSV	Non-specific protein target /polyclonal antibodies	-First therapy accepted by the FDA for human use. -Widely used treatment in the absence of other specific therapies	-Does not induce immunological memory. -High and recurrent doses are required to promote protection.	(Anderson et al. 1986; Groothuis et al. 1993; Respiratory Syncytial Virus (RSV) PREVENT study group 1997)
131-2G	G protein/ monoclonal antibody	-It is able to confer protection prior to or after hRSV-infection. -Triggers activated IFN-γ^+^ CD4^+^ and CD8^+^ T cells. -Widely used to identify an hRSV infection in laboratory assays. -Recognizes a very conserved epitope associated with the binding to its receptor.	-Does not induce immunological memory. -Not accepted by the FDA for human use. -Only approved in animal models.	(Tripp et al. 2001; Tripp et al. 2003; Radu et al. 2010; Miao et al. 2009; Haynes et al. 2009; Boyoglu-Barnum et al. 2014; Caidi et al. 2012; YOUNG 2002)
Palivizumab (MEDI 493)	F protein/ monoclonal antibody	-Decreases over 50% of neonatal hRSV-infection. -Accepted by the FDA for human use. -It is the only treatment used in humans nowadays. -Prevents the entry of the virus into the cell.	-Does not induce immunological memory. -At least 3 to 5 doses are necessary. -High cost (US$1416 dose of 100 mg/mL). -Difficult access for the high-risk population.	(Johnson et al. 1997; Subramanian et al. 1998; Sáez-Llorens et al. 1998; DeVincenzo et al. 2007; Village 1998; B. R. 2018; Torchin et al. 2018; Ambrose et al. 2014; Mochizuki et al. 2017; Lacaze-Masmonteil et al. 2003; Wu et al. 2007)
Motavizumab (MEDI 524)	F protein/ monoclonal antibody	-Decreases over 50% of neonatal infection. -Has higher affinity than palivizumab for its antigen. -Promotes a better protective effect than palivizumab. -Prevents the entry of the virus into the cell.	-Does not induce immunological memory. -At least 3 to 5 doses are necessary. -Not accepted by the FDA for human use. -Produces cutaneous lesions in human.	(Wu et al. 2008; Mejías et al. 2005; Huang et al. 2010; Fernández et al. 2010; Carbonell-Estrany et al. 2010; O’Brien et al. 2015; Ramilo et al. 2014; Mak et al. 2014)
Monoclonal anti-N	N protein/ monoclonal antibody	-High specificity in clinical samples from nasopharyngeal swabs from hRSV-infected patients. - May induce ADCC and complement fixed in infected cells. - N-hRSV protein migrates to the membrane of infected cells.	- The evaluation of this antibody is in experimental process in murine model	(Anderson et al. 1988; Aliprantis et al. 2018)

### Concluding remarks

Antibodies have been widely explored as a potent and recurrent strategy to prevent hRSV-infection in high-risk populations, especially due to the lack of an effective, safe, and licensed vaccine. Antibody-based approaches have been tested either as prophylactic or therapeutic treatments, with various results, depending on the antibody molecule evaluated. However, despite various efforts and several possible treatments, only one antibody is currently used to prevent the viral infection by hRSV, which is highly expensive and not always effective. For this reason, it is still essential to explore new options that could provide improved cost/effectiveness ratios, until a vaccine becomes available and allows the promotion of a protective immune response against hRSV.

## Data Availability

Not applicable.

## Abbreviations

hRSV: Respiratory Syncytial Virus
ALRTI: Acute Lower Respiratory Tract Infections
CNS: Central Nervous System
LRTI: Lower Respiratory Tract Infection
WHO: World Health Organization
NS: Non-structural protein
FI-hRSV: Formalin-inactivated hRSV vaccine
IVIG: Intravenous Immunoglobulin
IVIG-hRSV: Intravenous Immunoglobulin against hRSV
FDA: Food and Drug Administration
MEDI-493: Palivizumab
131-2G: G-hRSV monoclonal antibody
130-6D: G-hRSV monoclonal antibody
CCR: Central Conserved Region
PFU: Plaque Forming Unit
MEDI-524: Motavizumab
CDR: Complementary Determining Region
M/P: Motavizumab and then Palivizumab
P/M: Palivizumab and then Motavizumab
AE: Adverse effects
